The article "Differential expression of ANXA6, HSP27, PRDX2, NCF2, and TPM4 during uterine cervix carcinogenesis: diagnostic and prognostic value" was published in 2010. Journal: Br J Cancer.

# Differential expression of ANXA6, HSP27, PRDX2, NCF2, and TPM4 during uterine cervix carcinogenesis: diagnostic and prognostic value

**DOI:** 10.1038/sj.bjc.6605992

**Published:** 2010-11-30

**Authors:** M I Lomnytska, S Becker, I Bodin, A Olsson, K Hellman, A-C Hellström, M Mints, U Hellman, G Auer, S Andersson

**Affiliations:** 1 Department of Obstetrics and Gynecology, Institute for Clinical Science and Technology, CLINTEC, Karolinska University Hospital, Huddinge, Karolinska Institutet, Stockholm SE-14186, Sweden; 2 Unit of Cancer Proteomics, Department of Oncology and Pathology, Karolinska Institutet, Karolinska University Hospital, Stockholm SE-171 76, Sweden; 3 Department of Oncology and Pathology, Karolinska Institutet, Karolinska University Hospital, Stockholm SE-171 76, Sweden; 4 Department of Gynecologic Oncology, Radiumhemmet, Karolinska University Hospital, Stockholm SE-171 76, Sweden; 5 Department of Obstetrics and Gynecology, Karolinska University Hospital, Solna, Karolinska Institutet, SE-17176 Stockholm, Sweden; 6 Ludwig Institute for Cancer Research, Ltd, Uppsala University, Box 595, Uppsala SE-75124, Sweden; 7 Department of Oncology and Medical Radiology, Lviv National Medical University, Pekarska street, 69, Lviv 79010, Ukraine

**Keywords:** cervical cancer precursors, squamous cervical cancer, diagnostics, marker protein patterns, immunohistochemistry

## Abstract

**Background:**

Cytology-based diagnostics of squamous cervical cancer (SCC) precursor lesions is subjective and can be improved by objective markers.

**Methods:**

IHC-based analysis of ANXA6, HSP27, peroxiredoxin 2 (PRDX2), NCF2, and tropomyosin 4 (TPM4) during SCC carcinogenesis.

**Results:**

Expression of ANXA6, HSP27, PRDX2, and NCF2 in the cytoplasm of dysplastic cells increased from cervical intraepithelial neoplasia 2/3 (CIN2/3) to microinvasive cancer. Invasive SCC showed lower expression of TPM4 than CIN and normal epithelium. CIN2/3 with the highest sensitivity and specificity differed from normal epithelium by cytoplasmic expression of HSP27. Patients with cytoplasmic HSP27 expression in SCC deviating from that observed in normal epithelium had worse relapse-free (*P*=0.019) and overall (*P*=0.014) survival. Invasive SCC with the highest sensitivity and specificity differed from normal epithelium by expression of PRDX2 and TPM4 in the cytoplasm, from CIN2/3 by the expression of ANXA6 and TPM4 in the cytoplasm, and from microinvasive SCC by the expression of PRDX2 and ANXA6 in the cytoplasm. The number of sporadic ANXA6+ cells between the atypical cells increased from CIN2/3 to invasive SCC.

**Conclusion:**

Detection of expression changes of the proteins ANXA6, HSP27, PRDX2, NCF2, and TPM4 in SCC precursor lesions may aid current cytological and pathological diagnostics and evaluation of prognosis.

Cervical cancer (CC) is the second most commonly diagnosed cancer among women worldwide (Garcia *et al*, 2007). The introduction of cytology-based screening has reduced incidence of the most common squamous cell cervical carcinoma (SCC), but CC remains a major problem in the developing world.

The aetiological role of human papillomaviruses (HPVs) for CC and precursor lesions has been established (Wallin *et al*, 1999; Munoz *et al*, 2003; Castellsague, 2008; Zur Hausen, 2009). Persistent infection with HR-HPV and expression of the viral oncogenes E6 and E7 are critical for malignant transformation (Zur Hausen, 2009), making detection and monitoring of HR-HPV carriers upon primary detection of abnormal cervical cytology an attractive approach (Nobbenhuis *et al*, 1999; Brismar *et al*, 2009). However, more than half of patients with normal cervical histopathology demonstrate infection with HR-HPV although gain of the 3q26 chromosome region, where the human telomerase RNA gene (*hTERC*) is located, is an early event during CC carcinogenesis (Alameda *et al*, 2009; Andersson *et al*, 2009). Detection of hTERC amplification discriminates low- and high-grade squamous intraepithelial lesions and identifies patients with histologically confirmed cervical intraepithelial neoplasia (CIN) and SCC (Andersson *et al*, 2009).

In 1928, both Babés and Papanicolaou (Babés, 1928; Papanicolaou, 1928) described the potential for desquamated cell material from the uterine cervix to serve as a diagnostic tool for detection of CC. However, a high false-negative rate remains a major clinical problem today. The accuracy of Pap smear technique for early detection of CC and precursor lesions has been evaluated and the results varied with false-negative rates ranging from 5% to 40% (Näslund *et al*, 1986). When compared with conventional Pap smears, LBC showed neither higher sensitivity nor specificity for detection of CIN (Arbyn *et al*, 2008).

Correct diagnosis is important for choice of therapy and avoiding of under- and over-treatment. This indicates need for additional objective markers of CC precursors in cervical cytology material that can be detected by professionals or assessed through automated technology, and thus improve early diagnostics.

One promising approach in the search for new cancer markers is proteomics. Proteomics is used to analyse and identify differentially expressed proteins in tissue samples, and to validate their significance as disease markers (Kulasingam and Diamandis, 2008). Proteomics was used in several studies of CC markers to identify a number of differentially expressed proteins, but without analysing their potential diagnostic value (Bae *et al*, 2005; Choi *et al*, 2005; Zhu *et al*, 2009). We previously used proteomics analysis to compare SCC and squamous vaginal cancer (Hellman *et al*, 2004, 2009; Lomnytska *et al*, 2010), and we extend the analysis in a current study aiming to establish a marker protein pattern for objective detection of SCC precursor lesions. We performed an analysis of expression of ANXA6, HSP27, peroxiredoxin 2 (PRDX2), NCF2, and tropomyosin 4 (TPM4) on sequential steps of SCC carcinogenesis, that is, on CIN2/3, microinvasive, and invasive cancers. We evaluated cytoplasmic and nuclear expression of these proteins in differentiated, dysplastic, and cancer cells, compared expression of proteins, and discussed the potential clinical value of the differential expression of the studied marker protein patterns.

## Materials and methods

### Clinical material

The study was performed on formaldehyde-fixed paraffin-embedded material, collected at the Department of Gynecology, Karolinska University Hospital, Huddinge, Sweden, and at the Department of Oncology and Medical Radiology, Lviv National Medical University, Ukraine with informed consent and approval from the local ethics committees (Stockholm County Council – Dnr. 97-244, 00-068, 352/00; Ethics Committee of Lviv National Medical University – protocol No. 2; Table 1A). Histopathological presentation of selected cases was confirmed.

### IHC

Paraffinised tissue blocks were cut to obtain 4 *μ*m-thick tissue sections on SuperFrost (Braunschweig, Germany) slides and kept overnight at 55°C before deparaffinisation and rehydratation that was carried out in a series of xylene and ethanol baths of decreasing concentration. Antigen was retrieved by boiling in 0.1 M Na citrate buffer (pH 6.0). Endogenous peroxidase was inhibited by 0.5% H_2_O_2._ Samples were incubated in 5% serum of the species from which the secondary antibody was obtained to avoid non-specific binding. Monoclonal antibodies to ANXA6 (1 : 400), PRDX2 (1 : 100), HSP27 (1 : 400), NCF2 (1 : 150), TPM4 (1 : 100), vimentin (1 : 200, V5255, Sigma-Aldrich, St Louis, MO, USA), and CD68 (1 : 400, PG-M1, DAKO, Carpinteria, CA, USA) in 1% BSA were applied and incubated overnight at +4°C (Table 1B). The secondary antibody was coupled to DAB via a biotin–avidin complex for visualisation (VectaStain, Vector, Burlingame, CA, USA). Tissue samples were counterstained with hematoxylin, washed in lukewarm water, dehydrated in a series of increasing concentrations of ethanol and xylene, mounted using a permanent mounting medium, and covered. All steps were carried out in a moist chamber.

### Evaluation of staining

Images were captured at a Leica DM4500B light microscope (camera DFC320, ocular 10 × , objectives 20 × /0.50 HC PL, and 40 × , 506145, Leica Application Suite software (version 2.4.0, Wetzlar, Germany), 16-bit depth.tif format images with 48bit/*μ*m image resolution). Expression of the analysed proteins was scored based on the intensity of staining, location of staining in individual cells, and on the number of positively stained cells. Intensity of colour expression was scored as: 0, negative; 1+, weak; 2+, moderate; and 3+, strong. The number of positively stained cells was scored as 0 if no staining was observed or was present in <5% of cells; 1+, positive staining in 5–25% of cells; 2+, positive staining in 25–75% of cells; and 3+, positive staining in more than 75% of cells. Expression of a protein was evaluated as a histoscore, that is, as a sum of the scores of the intensity and of the cell number counts (Cheng *et al*, 2008).

### DNA cytometry

DNA cytometry was performed on tissue sections (6 *μ*m) of CIN2/3 and SCC. Slides were stained with Feulgen and the DNA content in nuclei of atypical cells was measured as described (Steinbeck *et al*, 1999). DNA values were determined in relation to a corresponding control, which denoted the normal DNA (diploid) content at 2c region. Histograms with a narrow stem line in the 2c region represented diploid genomically stable tumours, whereas those with a broad stem line in the 2c region expanding towards the 4c region were classified as diploid genomically unstable. Histograms with a narrow peak outside the 2c region were considered to be aneuploid genomically stable, whereas with a broad peak outside the 2c region and additional peaks exceeding the 4c region were classified as aneuploid genomically unstable. Approximately 100 cells were analysed for each tumour specimen.

### Statistical analysis

Software Statistica 6.0 (StatSoft Inc., Tulsa, OK, USA) was used for the *χ*^2^ test, *t*-test, *P*-value, software MedCalc 11.2.1.0 (MedCalc Software bvba, Mariakerke, Belgium) for ROC analysis, evaluation of sensitivity and specificity. Relapse-free survival (RFS) and overall survival (OS) were evaluated using univariate Kaplan–Meier analysis with log-rank test. A difference of *P*<0.05 was considered statistically significant (Glantz, 1998).

## Results

### Intensity of expression of ANXA6, HSP27, PRDX2, NCF2, and TPM4 in normal uterine cervix and during development of SCC

In squamous cervical epithelial (*SCE*), expression of ANXA6 was localised to the epithelial cell membrane with moderately intense expression in the submucosal stroma. Positive expression of HSP27, PRDX2, NCF2, and TPM4 was observed in the cytoplasm (Figure 1; Table 2A).

In *CIN2,* we observed weak and moderate expression of ANXA6 in the cytoplasm of dysplastic cells; parabasal cells were characterised by moderate cytoplasmic protein expression. Additionally, we observed strong expression of ANXA6 in 5 to 10% of cells within the dysplastic cell layer. Those cells were negative for expression of vimentin (VIM−) and CD68. Strong cytoplasmic expression of HSP27 and its stromal expression were detected. NCF2 and TPM4 showed weak cytoplasmic expression.

In *CIN3,* dysplastic cells showed weak and moderate expression of ANXA6 in 18 cases (72%) with a presence of sporadic ANXA6+ cells. Weak and moderate nuclear expression of HPS27 was detected in addition to moderate/strong cytoplasmic and stromal expression. Peroxiredoxin 2 was positive in only one out of three cases, NCF2 in half of cases, and TPM4 in two out of three cases. In CIN2/3, NCF2+ cells were localised to the deep parabasal layers of epithelium, and TPM4+ cells were seen in superficial differentiated layers.

In *MicSCC,* expression of ANXA6 was positive in cancer cells in seven (77.8%) cases showing presence of sporadic ANXA6+ cells. Expression of HSP27 was predominantly cytoplasmic moderate. Peroxiredoxin 2 and NCF2 were positive in almost all cases, whereas TPM4 was detected in five (55.6%) cases.

In *InvSCC,* sporadic ANXA6+ cells (5–30%) were observed in 19 (79.2%) cases, although diffuse cytoplasmic expression of the protein was uncommon. Moderate/strong cytoplasmic expression of HSP27 was found in almost all cases and moderate nuclear expression in half the cases (11–43.8%). Weak cytoplasmic expression of PRDX2 and NCF2 was observed. Weak cytoplasmic expression of TPM4 was found in six (25%) cases.

### Histoscore of expression of ANXA6, HSP27, PRDX2, NCF2, and TPM4 in SCC carcinogenesis

The histoscore (a sum of scores representing number of cells expressing the protein and intensity of staining) is another parameter used to evaluate proteins. Diffuse cytoplasmic expression of ANXA6 was lower in InvSCC than in MicSCC and CIN3. The number of sporadic ANXA6+ cells increased towards InvSCC (Figure 2; Table 2B). Expression of HSP27 in the cytoplasm of dysplastic cells was higher in CIN2/3 than in SCE. A diffuse cytoplasmic expression of NCF2 was similar in the dysplastic cells of CIN2/3, but higher in MicSCC than in InvSCC. Expression of PRDX2 in MicSCC was similar to expression in SCE, which was higher than in InvSCC. Tropomyosin 4 expression in the cytoplasm of dysplastic and cancer cells gradually decreased from SCE to InvSCC, with a significant difference between CIN3 and InvSCC.

### Sensitivity and specificity

For distinguishing between normal SCE and CIN2/3, expression of HSP27 in the cytoplasm had the best sensitivity and specificity (Figure 3A). Expression of PRDX2 and TPM4 in the cytoplasm was associated with both the highest sensitivity and specificity for differentiation between SCE and InvSCC, and expression of PRDX2 and ANXA6 in the cytoplasm was the most sensitive and specific for differentiation between MicSCC and InvSCC (Figure 3B). Finally, expression of ANXA6 and TPM4 in the cytoplasm provided the best specificity and sensitivity for distinguishing between CIN2/3 and InvSCC.

### Coexpression of ANXA6, HSP27, PRDX2, NCF2, and TPM4 in CIN3 and SCC

ANXA6 was coexpressed with PRDX2 in the cytoplasm of dysplastic cells in 3/4 of cases (*P*=0.057; Table 3) of CIN3 and MicSCC. A correlation between genomic instability and positive nuclear expression of HSP27 in dysplastic cells was observed. Between genomically unstable CIN2/3 and MicSCC, 11 (91.7%) cases with positive nuclear expression of HSP27 (*P*=0.061) were found.

### Prognostic value of cytoplasmic HSP27 expression in InvSCC cancer cells

Relapse-freeRFS and OS were evaluated in 14 patients with InvSCC, who were followed for 60–72 months (5–6 years) after primary diagnosis (Figure 4C). Patients with weak HSP27 cytoplasmic expression (two cases, 14.3%) had the worst RFS (*P*=0.019) and OS (*P*=0.014), compared with other patients (Figure 4A and B). Patients with strong HSP27 cytoplasmic expression (four cases, 28.6%) had worse RFS (*P*=0.062) and OS (*P*=0.048) than patients with moderate expression of that protein (eight cases, 57.1%). Among the nine patients who were diagnosed at stages IB1-2, three patients showed strong HSP27 expression, whereas six patients showed moderate expression of the protein. Within a 3–4-year period, relapse with lethal outcome was observed in two (66.7%) out of three cases with strong HSP27 expression and in one (16.7%) out of six cases with moderate protein expression (*P*<0.001).

## Discussion

Mutations that occur during progression from dysplasia to invasive SCC are reflected by changes in expression of tissue proteins. We previously identified the differential protein marker pattern that characterises SCC (Hellman *et al*, 2009; Lomnytska *et al*, 2010), and in current study, we analysed expression of proteins ANXA6, HSP27, PRDX2, NCF2, and TPM4 during SCC carcinogenesis.

We observed that ANXA6 expression gradually increased during the progression from CIN2 to MicSCC, whereas it decreased in InvSCC. Cleavage of the NH_2_-domain severely impairs the function of ANXA6 (Gerke and Moss, 2002), while full-length ANXA6 is generally described to be under expressed in cancer and during carcinogenesis (Francia *et al*, 1996). Previously, we found that only the NH_2_-terminal domain of ANXA6 was overexpressed in SCC (Lomnytska *et al*, 2010), which may indicate dysfunction of ANXA6 in SCC and explain the decrease in expression of full-length protein, as detected by IHC in cases of InvSCC. ANXA6 localises to the endoplasmic reticulum and plasma membrane (Barwise and Walker, 1996), and relocation of the protein from the cytosol to the plasma membrane is dependent on the elevation of Ca^2+^ influx (Buzhynskyy *et al*, 2009; Sztolsztener *et al*, 2009). We did not observe ANXA6 expression on plasma membranes of atypical cells, where expression was mainly cytoplasmic. One regulator of ANXA6-dependent plasma membrane dynamics is EGF, through the EGF-dependent influx of Ca^2+^ (Strzelecka-Kiliszek *et al*, 2008), and development of CC is also determined by EGF activity (Bellone *et al*, 2007). We observed that the number of strongly ANXA6+ cells increased during the progression from CIN2 to InvSCC. We previously suggested that this observation represents nuclear expression of ANXA6 in cancer cells (Lomnytska *et al*, 2010), however, because of the variable histopathological appearance we could not exclude the possibility that these were infiltrating immune cells. Further analysis showed that these cells were negative for vimentin and CD68 and thus could not be identified as fibroblasts, endothelial cells, lymphoid cells, monocytes, or macrophages. Appearance of ANXA6+ cells only between dysplastic and cancer cells was an interesting observation, which may improve diagnosis.

HSP27 is a member of the HSP family that maintains protein structure, restores denaturated, aggregated, and damaged proteins, and are therefore activates when subjected to different types of stress, such as oxidative stress, inflammation, and malignant transformation (Ciocca and Calderwood, 2005). It was recently reported that HSP27 expression in cervical precursor lesions is higher than in SCE, and that it is higher in invasive SCC than in precursor lesions (Ono *et al*, 2009). We have also observed increase of the cytoplasmic expression of HSP27 in cervical precursor lesions. However, cytoplasmic expression of HSP27 in microinvasive and invasive SCC was lower than in precursor lesions. Previously noted low sporadic expression or no expression of HSP27 in InvSCC was not explained (Ono *et al*, 2009). We observed that RFS and OS for patients with weak or strong HSP27 expression in cancer cells were lower than for patients with moderate and essentially normal (as in SCE) protein expression. In uterine cervix, HSP27 has a role in the maturation of squamous cells and is associated with more differentiated tumours, whereas its decreased expression associates dedifferentiation and transformation to adenocarcinoma. At the same time, highly expressed HSPs, including HSP27, may facilitate cancer progression by repairing cells that were damaged by chemo- and radiotherapy and by protecting them from apoptosis (Ciocca and Calderwood, 2005). CIN2/3, microinvasive, and invasive SCC were characterised by nuclear expression of HSP27. In eukaryotic cells, HSPs and HSP27 relocate to nuclei under stress, whereas HSP27 is found to be a permanent component of the interchromatin granule clusters known as nuclear speckles (Van den IJssel *et al*, 2003). We observed a link between positive nuclear expression and genomic instability in CIN2/3 and MicSCC. It was shown that in cervical smears the number of cells with genomic instability gradually increase during the progression from low- to high-grade intraepithelial lesions (Singh *et al*, 2008). Development of chromosomal instability is the initial consequence of HPV infection, representing a preparatory event in the integration of the virus into the genome (Melsheimer *et al*, 2004). Finally, HPV has an influence on HSP27 expression (Ciocca and Calderwood, 2005).

Peroxiredoxins have been linked with regulation of proliferation, differentiation, and apoptosis (Park *et al*, 2006). Peroxiredoxin 2 has both proliferative and antiapoptotic properties and thus may induce carcinogenic changes (Noh *et al*, 2001). When overexpressed, PRDX2 protects cancer cells from oxidative stress and thus mediates resistance to chemo- and radiotherapy (Soini *et al*, 2006; Smith-Pearson *et al*, 2008). NCF2 is an NADPH oxidase cytosolic component and the gene that encodes this protein is upregulated by TNF-*α* (Gauss *et al*, 2005; Ammons *et al*, 2007). TNF-*α* and the encoding gene impact development of CC by increasing susceptibility to infection with HR-HPV (Deshpande *et al*, 2005). In our study, NCF2 was overexpressed in MicSCC. In cervical precursor lesions, we observed a tendency for coexpression of ANXA6 and NCF2.

Tropomyosins (TPMs) are actin-interacting protein components of the cytoskeleton that have been implicated in neoplastic-specific alterations of actin-based organisation. Rearrangement of microfilament bundles, morphological alterations, and increased cell motility are major features of a transformed phenotype and are usually associated with decreased expression of nonmuscle isoforms of TPMs (Helfman *et al*, 2008). Decreased expression of TPMs can be caused by hypermethylation of the encoding gene (Bharadwaj and Prasad, 2002) or dysfunction of Rho-kinase (Bharadwaj *et al*, 2005). In our study, expression of the TPM4 protein was significantly lower in MicSCC and InvSCC than in precancerous lesions and SCE. In precursor lesions we observed coexpression of TPM4 and NCF2, usually characterised by overexpression of NCF2 in atypical cells and of TPM4 in differentiated cells.

Our study is the first to assess a marker proteins pattern previously identified by proteomics-based analysis of SCC for the changes in expression during the sequential steps of SCC carcinogenesis. In particular, cytoplasmic expression of ANXA6 gradually increased in CIN and MicSCC and decreased in InvSCC. Sporadic ANXA6+ cells were observed between dysplastic cells. Cytoplasmic expression of HSP27 increased towards CIN and was more intense in dysplastic lesions than in MicSCC and InvSCC. Cervical precursor lesions and invasive cancer were characterised by nuclear expression of HSP27. MicSCC was characterised by overexpression of PRDX2 and NCF2, whereas expression of TPM4 was observed mostly in SCE and partially in precursor lesions. Our findings describing the differences in expression of marker proteins during SCC carcinogenesis may be useful for developing more objective methods for early diagnosis of precursor SCC lesions and for monitoring patients.

## Figures and Tables

**Figure 1:** Six selected cases (1–6) showing immunohistochemical expression of ANXA6 (**A**), HSP27 (**B**), PRDX2 (**C**), NCF2 (**D**), and TPM4 (**E**), magnification: × 400 (**D1**, **D2**, **E2**, **C6** have magnification × 200), noncropped images with inserts. Observed expression of ANXA6 was membranous in SCE (**A1**), cytoplasmic and sporadic in CIN2/3, MicSCC and InvSCC (**A2**–**A6**). Expression of HSP27 in the nuclei was observed in CIN2/3, MicSCC (**B2**–**B4**), and less in InvSCC (**B5**–**B6**). Expression of PRDX2 was cytoplasmic in positive cases. Expression of NCF2 was observed in the cytoplasm (**D2**–**D6**), and expression of TPM4 in the cytoplasm was observed mainly in SCE (**D1**). Histopathological description. SCE (1): stratified layers of epithelial cells with a thin layer of parabasal cells. CIN2/3 (2–3): dysplastic cells with hyperchromatic irregular nuclei and koilocytar atypia with perinuclear clear vacuolisation as characteristic of HPV infection (marked with black arrows – **C2**, **A4**, **B4**) that gradually substitute epithelial layers from basal membrane throughout the epithelium forming carcinoma *in situ*. MisSCC (4): invasion of dysplastic cells into underlying stroma for <3 mm in depth and <7 mm horizontally. InvSCC (5–6): irregular infiltrates of tumor cells in connective tissue with inflammatory reaction.

**Figure 2:** Changes in the expression of ANXA6 (**A**), HSP27 (**B**), NCF2, and TPM4 (**C**) during SCC carcinogenesis. Compared histoscores are presented in Table 2B, polynomial trend lines of the corresponding colour that depict changes in the expression of proteins. Significantly different values (*t*-test, *P*<0.05) of corresponding colour are marked by ^*^, †, ‡ for the corresponding colour; ^§^*P*=0.085.

**Figure 3:** ROC curves displaying sensitivity and specificity for detection of CIN2/3 by expression of HSP27 (**A**), differentiation of MicSCC from InvSCC (**B**), and of CIN2/3 from MicSCC and InvSCC by expression of ANXA6, PRDX2, TPM4, HSP27, and NCF2 in the cytoplasm (**C**). Cutoff for histoscores is presented in corresponding tables.

**Figure 4:** Relapse-free (**A**) and overall (**B**) survival of patients with SCC (**C**) with various expression of HSP27 in cytoplasm of cancer cells (univariate method by Kaplan–Meier, log-rank test).

**Table 1:** Characterisation of clinical material (A) and primary antibodies used for immunohistochemistry (IHC) (B)

**(A)**			
**Diagnosis, FIGO**	**Histopathology**	**Abbrevation**	**Number of cases (%)**
Normal cervix	Normal cervix	SCE	8 (11.94)
CIN 2	Moderate cervical intraepithelial dysplasia	CIN 2	4 (5.97)
CIN 3	Severe cervical intraepithelial dysplasia	CIN 3	9 (13.43)
	Squamous cervical carcinoma *in situ*		12 (17.91)
SCC, stage IA1	Microinvasion <3 mm in depth and <7 mm horizontally	MicSCC	7 (10.45)
SCC, stage IA2	Invasion >5 mm in depth or >7 mm horizontally	InvSCC	2 (2.99)
SCC, stage IB1	Visible lesion ≤4 cm in greatest dimension		17 (25.37)
SCC, stage IB2	Visible lesion >4 cm		2 (2.99)
SCC, stage IIA	Without parametrial invasion, but involvimg upper 2/3 of vagina		1 (1.49)
SCC, stage IIB	With parametrial invasion		1 (1.49)
SCC, stage III	Extends to pelvic wall or lower third of vagina		3 (4.48)
Total			66

**(B)**							
**Protein**	**Antibody**	**Origin**	**Clone**	**Epitope detection**	**Dilution factor**	**Tissues for positive controls**	**Manufacturer**
ANXA6	Sc-1931	Goat polyclonal	N-19	N-terminus	400	Liver hepatocytes	SantaCruz (SantaCruz, CA, USA)
HSP27	Sc-13132	Mouse monoclonal	F-4	Amino acids 32–108	400	Tonsilla	SantaCruz (SantaCruz, CA, USA)
PRDX2	WH007001	Mouse monoclonal	4E 10-2D2	Amino acids 1–199	100	Tonsilla	Sigma-Aldrich
NCF2	HPA006040	Rabbit polyclonal	PrEST	Full-length	150	Glandular epithelium of colon	Sigma-Aldrich
TPM4	WH000717	Mouse monoclonal	4E4-1D2	Full-length	200	Placenta, decidual tissue	Sigma-Aldrich

Abbreviations: CIN=cervical intraepithelial neoplasia; FIGO=International Federation of Gynecologic Oncology; SCC=squamous cervical cancer; SCE=squamous cervical epithelial.

**Table 2:** Breakdown of studied cases by intensity of expression of ANXA6, HSP27, PRDX2, NCF2, and TPM4 (A) and histoscore (B)

**(A)**																			
	**Breakdown of cases by the intensity of expression of protein, number of patients (%)**																		
	**ANXA6, cytoplasmic expression**				**ANXA6, sporadic cells**				**HSP27, cytoplasmic expression**				**HSP27, nuclear expression**				**HSP27, stroma**		
**Diagnosis**	**0**	**1+**	**2+**	**3+**	**0**	**1+**	**2+**	**3+**	**0**	**1+**	**2+**	**3+**	**0**	**1+**	**2+**	**3+**	**0**	**1+**	**2+**
SCE	0	0	0	0	0	0	0	0	0	0	8 (100.0)	0	0	0	0	0	5 (62.5)	3 (36.5)	0
CIN2	3 (42.8)	2 (28.6)	2 (28.6)	0	1 (25)	0	0	3 (75.0)	0	0	1 (25.0)	3 (75.0)	2 (50.0)	1 (25.0)	1 (25.0)	0	1 (25.0)	0	3 (75.0)
CIN3	7 (28.0)	9 (36.0)	9 (36.0)	0	9 (36)	0	0	16 (64.0)	0	0	8 (32.0)	17 (68.0)	11 (44.0)	7 (28.0)	7 (28.0)	0	11 (45.8)	4 (16.7)	9 (37.5)
MicSCC	2 (22.2)	3 (33.3)	4 (44.4)	0	2 (25)	0	1	6 (75)	0	0	5 (62.5)	3 (37.5)	5 (62.5)	0	3 (37.5)	0	7 (77.8)	2 (22.2)	0
InvSCC	18 (75)	4 (16.7)	2 (8.3)	0	2 (8.3)	0	3 (12.5)	19 (79.2)	0	2 (8.3)	15 (62.5)	7 (29.2)	13 (54.2)	0	10 (41.7)	1 (4.2)	15 (62.5)	9 (37.5)	0
																			
	**PRDX2, cytoplasmic expression**				**NCF2, cytoplasmic expression**				**NCF2, sporadic cells**				**NCF2, stroma**				**TPM4, cytoplasmic expressiom**		
	**0**	**1+**	**2+**	**3+**	**0**	**1+**	**2+**	**3+**	**0**	**1+**	**2+**	**3+**	**0**	**1+**	**2+**	**3+**	**0**	**1+**	
SCE	1 (20.0)	4 (80.0)	0	0	4 (50.0)	4 (50.0)	0	0	0	0	0	0	0	0	0	0	1 (12.5)	7 (87.5)	
CIN2	—	—	—	—	1 (25.0)	3 (75.0)	0	0	3 (75)	0	0	1 (25.0)	3 (75.0)	0	0	1 (25.0)	1 (25.0)	3 (75.0)	
CIN3	7 (63.3)	4 (36.4)	0	0	11 (44.0)	14 (56.0)	0	0	11 (84.6)	0	1 (7.7)	1 (7.7)	11 (84.6)	0	0	2 (15.4)	7 (28.0)	18 (62.0)	
MicSCC	0	7 (100)	0	0	2 (22.2)	7 (77.8)	0	0	0	0	0	0	0	0	0	0	4 (44.4)	5 (55.6)	
InvSCC	8 (80.0)	2 (20.0)	0	0	17 (70.8)	6 (25)	1 (4.2)	0	9 (37.5)	0	10 (41.7)	5 (20.8)	20 (86.9)	1 (4.3)	2 (8.6)	0	18 (75)	6 (25)	

**(B)**																				
	ANXA6*				HSP27*						PRDX2*		NCF2*						TPM4*	
	**Cytoplasmic**				**Cytoplasm**		**Nuclear**		**Stromal**		**cytoplasmic**		**Cytoplasmic**				**Stromal**	**Cytoplasmic**		
**Diagnosis**	**Diffuse**	***P*-value**	**Sporadic**	***P*-value**		***P*-value**		***P*-value**		***P*-value**		***P*** **-value**	**Diffuse**	***P*** **-value**	**Sporadic**	***P*** **-value**		***P*** **-value**		***P*** **-value**
SCE	0		0		5.0±0	1, 3	0		1.5±2.07	1, 3	3.2±1.79	1	1.63±1.77	1, 2	0		0		3.38±1.41	2
CIN 2	2.25±2.63	1	2.25±1.50	1	5.75±0.50	1, 2	2.25±2.63	1	3.75±2.50	1, 2	—		2.75±1.89	1	0.5±1.0	1	0.75±1.50	1	3.0±2.0	1
CIN 3	3.33±2.03	1, 2, 3	1.86±1.49	1, 2, 3	5.67±0.48	2, 3, 4	2.10±1.97	1, 2, 3	2.30±2.39	2, 3, 4	1.50±1.92	1, 2	1.90±1.92	2, 3	0		0		2.52±1.78	1, 2, 3
MicSCC	3.56±2.07	2, 4	2.56±1.67	2	5.38±0.52		1.75±2.43	2	0.89±1.76		4.0±0	2, 3	3.11±1.76	3, 4	0		0		2.22±2.11	4
InvSCC	1.08±1.93	3, 4	2.71±1.16	3	5.21±0.53	4	1.83±2.18	3	1.5±1.98	4	0.8±1.69	3	1.21±1.93	4	1.46±1.35	1	0.75±1.73	1	0.96±1.71	3, 4
*P-*value	0.358754	1	0.634305	1	**0.00119**	1	0.892191	1	0.12707	1	0.11240458	1	0.3330842	1	0.188829	1	1	1	0.633935	1
	0.786863	2	0.266001	2	0.755778	2	0.695733	2	0.28235	2	**0.003522**	2	0.7233573	2					0.23591	2
	**0.00045**	3	**0.0373**	3	**0.00064**	3	0.676471	3	0.41439	3	**0.000168**	3	0.1180145	3					**0.00435**	3
	**0.00305**	4			**0.00703**	4			0.23065	4			**0.015041**	4					**0.0852**	4

Abbreviations: CIN=cervical intraepithelial neoplasia; InvSCC=invasion SCC; MicSCC=microinvasion SCC; SCC=squamous cervical cancer; SCE=squamous cervical epithelial.

^*^ Histoscore: score of the intensity of expression plus the score of the number of cells that express the protein. Bold values stand for statistically significant differences.

**Table 3:** Coexpression of proteins in CIN3, microinvasive and invasive SCC

			**Protein 2, localisation**		
			**ANXA6, cyt**		
**Diagnosis**	**Protein 1, localisation**		**Positive**	**Negative**	***P*-value**
CIN 3 – MicSCC	PRDX2, cyt	Positive	12/18 (66.7%)	0/2	*0.057*
	(*n*=20)	Negative	5/18 (27.8%)	2/2 (100%)	
	TPM4, cyt	Positive	16/24 (66.7%)	2/5 (40%)	0.272
	(*n*=29)	Negative	8/24 (33.3%)	3/5 (60%)	
	NCF2, cyt	Positive	15/23 (65.2%)	2/5 (40%)	0.304
	(*n*=28)	Negative	8/23 (34.7%)	3/5 (60%)	
InvSCC	NCF2, cyt	Positive	2/6 (33.3%)	6/20 (30%)	0.879
					
	(*n*=26)	Negative	4/6 (66.7%)	14/20 (70%)	
					
			**NCF2, cyt**		
CIN 3 – MicSCC	TPM4, cyt	Positive	9/11 (81.8%)	6/10 (60%)	0.281
	(*n*=21)	Negative	2/11 (18.2%)	4/10 (40%)	
	HSP27, nuc	Positive	7/10 (70%)	5/10 (50%)	0.222
	(*n*=20)	Negative	2/10 (20%)	5/10 (50%)	
					
InvSCC	TPM4, cyt	Positive	2/8 (25%)	6/18 (33.3%)	0.677
	(*n*=26)	Negative	6/8 (75%)	12/18 (66.7%)	
	HSP27, nuc	Positive	6/8 (75%)	7/18 (38.9%)	*0.096*
	(*n*=26)	Negative	2/8 (25%)	11/18 (61.1%)	
					
			**HSP27, nuc**		
CIN 3 – MicSCC	TPM4, cyt	Positive	9/12 (75%)	5/8 (62.5%)	0.560
	(*n*=20)	Negative	3/12 (25%)	3/8 (37.5%)	
	Ploidy	DAU*	11/12 (91.7%)	5/9 (55.6%)	*0.061*
	(*n*=21)	DAS*	1/12 (8.3%)	4/9 (43.4%)	
					
InvSCC	TPM4, cyt	Positive	4/12 (33.3%)	3/12 (25%)	0.66
	(*n*=24)	Negative	8/12 (66.7%)	9/12 (75%)	
	Ploidy	DAU*	10/12 (83.3%)	13/13 (100%)	*0.133*
	(*n*=25)	DAS*	2/12 (16.7%)	0/13	
					
			**NCF2, sporadic**		
InvSCC	ANXA6, sporadic	Positive	14/15 (93.3%)	16/18 (88.9%)	0.663
	(*n*=33)	Negative	1/15 (6.7%)	2/18 (11.1%)	

Abbreviations: CIN=cervical intraepithelial neoplasia; InvSCC=invasion SCC; MicSCC=microinvasion SCC; PRDX=peroxiredoxin; SCC=squamous cervical cancer; TPM=tropomyosin. ^*^DAU=diploid and aneuploid unstable; ^*^DAS-diploid and aneuploid stable.

## References

[bib1] Alameda F, Espinet B, Corzo C, Munoz R, Bellosillo B, Lloveras B, Pijuan L, Gimeno J, Salido M, Sole F, Carreras R, Serrano S (2009) 3q26 (hTERC) gain studied by fluorescence *in situ* hybridization as a persistence-progression indicator in low-grade squamous intraepithelial lesion cases. Hum Pathol 40: 1474–14781954055710.1016/j.humpath.2009.03.013

[bib2] Ammons MC, Siemsen DW, Nelson-Overton LK, Quinn MT, Gauss KA (2007) Binding of pleomorphic adenoma gene-like 2 to the tumor necrosis factor (TNF)-alpha-responsive region of the NCF2 promoter regulates p67(phox) expression and NADPH oxidase activity. J Biol Chem 282: 17941–179521746299510.1074/jbc.M610618200

[bib3] Andersson S, Sowjanya P, Wangsa D, Hjerpe A, Johansson B, Auer G, Gravitt PE, Larsson C, Wallin K-L, Ried T, Heselmeyer-Haddad K (2009) Detection of genomic amplification of the human telomerase gene TERC, a potential marker for triage of women with HPV-positive, abnormal Pap smears. Am J Pathol 175: 1831–18471988082610.2353/ajpath.2009.090122PMC2770709

[bib4] Arbyn M, Bergeron C, Klinkhamer P, Martin-Hirsch P, Siebers AG, Bulten J (2008) Liquid compared with conventional cervical cytology: a systematic review and meta-analysis. Obstet Gynecol 111: 167–1771816540610.1097/01.AOG.0000296488.85807.b3

[bib5] Babés A (1928) Cancer du col uterin par Les-Frottis. Presse Med 29: 451

[bib6] Bae SM, Lee CH, Cho YL, Nam KH, Kim YW, Kim CK, Han BD, Lee YJ, Chun HJ, Ahn WS (2005) Two-dimensional gel analysis of protein expression profile in squamous cervical cancer patients. Gynecol Oncol 99: 26–351605132910.1016/j.ygyno.2005.05.041

[bib7] Barwise JL, Walker JH (1996) Annexins II, IV, V and VI relocate in human foreskin fibroblasts. J Cell Sci 109: 247–255883480910.1242/jcs.109.1.247

[bib8] Bellone S, Frera G, Landolfi G, Romani C, Bandiera E, Tognon G, Roman JJ, Burnett AF, Pecorelli S, Santin AD (2007) Overexpression of epidermal growth factor type-1 receptor (EGF-R1) in cervical cancer: implications for Cetuximab-mediated therapy in recurrent/metastatic disease. Gynecol Oncol 106: 513–5201754043710.1016/j.ygyno.2007.04.028

[bib9] Bharadwaj S, Prasad GL (2002) Tropomyosin-1, a novel suppressor of cellular transformation is downregulated by promoter methylation in cancer cells. Cancer Lett 26: 205–21310.1016/s0304-3835(02)00119-212065096

[bib10] Bharadwaj S, Thanawala R, Bon G, Falcioni R, Prasad GL (2005) Resensitization of breast cancer cells to anoikis by tropomyosin-1: role of Rho kinase-dependent cytoskeleton and adhesion. Oncogene 15: 8291–830310.1038/sj.onc.120899316170368

[bib11] Brismar S, Johansson B, Borjesson M, Arbyn M, Andersson S (2009) Follow-up after treatment of cervical intraepithelial neoplasia by human papillomavirus genotyping. Am J Obstet Gynecol 201: 17e1–17e81934488110.1016/j.ajog.2009.01.005

[bib12] Buzhynskyy N, Golczak M, Lai-Kee-Him J, Lambert O, Tessier B, Gounou C, Bérat R, Simon A, Granier T, Chevalier JM, Mazères S, Bandorowicz-Pikula J, Pikula S, Brisson AR (2009) Annexin-A6 presents two modes of association with phospholipid membranes: a combined QCM-D, AFM and cryo-TEM study. J Struct Biol 168: 107–1161930692710.1016/j.jsb.2009.03.007

[bib13] Castellsague X (2008) Natural history and epidemiology of HPV infection and cervical cancer. Gynecol Oncol 110: S4–S71876071110.1016/j.ygyno.2008.07.045

[bib14] Cheng AL, Huang WG, Chen ZC, Zhang PF, Li MY, Li F, Li JL, Li C, Yi H, Peng F, Duan CJ, Xiao ZQ (2008) Identificating cathepsin D as a biomarker for differentiation and prognosis of nasopharyngeal carcinoma by laser capture microdissection and proteomic analysis. J Proteome Res 7: 2415–24261843315510.1021/pr7008548

[bib15] Choi YP, Kang S, Hong S, Xie X, Cho NH (2005) Proteomic analysis of progressive factors in uterine cervical cancer. Proteomics 5: 1481–14931583890210.1002/pmic.200401021

[bib16] Ciocca DR, Calderwood SK (2005) Heat shock proteins in cancer: diagnostic, prognostic, predictive, and treatment implications. Cell Stress Chaperones 10: 86–1031603840610.1379/CSC-99r.1PMC1176476

[bib17] Deshpande A, Nolan JP, White PS, Valdez YE, Hunt WC, Peyton CL, Wheeler CM (2005) TNF-alpha promoter polymorphisms and susceptibility to human papillomavirus 16-associated cervical cancer. J Infect Dis 191: 969–9761571727410.1086/427826

[bib18] Francia G, Mitchell SD, Moss SE, Hanby AM, Marshall JF, Hart IR (1996) Identification by differential display of annexin-VI, a gene differentially expressed during melanoma progression. Cancer Res 56: 3855–38588752144

[bib19] Garcia M, Lemal A, Ward EM, Center MM (2007) Global cancer facts and figures. American Cancer Society: Atlanta, GA

[bib20] Gauss KA, Bunger PL, Larson TC, Young CJ, Nelson-Overton LK, Siemsen DW, Quinn MT (2005) Identification of a novel tumor necrosis factor alpha-responsive region in the NCF2 promoter. J Leukoc Biol 77: 267–2781551396710.1189/jlb.0604329

[bib21] Gerke V, Moss SE (2002) Annexins: from structure to function. Physiol Rev 82: 331–3711191709210.1152/physrev.00030.2001

[bib22] Glantz S (1998) Medico-Biological Statistics. Medicyna Praktika: Moscow, 128p

[bib23] Helfman DM, Flynn P, Khan P, Saeed A (2008) Tropomyosin as a regulator of cancer cell transformation. Adv Exp Med Biol 644: 124–1311920981810.1007/978-0-387-85766-4_10

[bib24] Hellman K, Alaiya AA, Becker S, Lomnytska M, Schedvins K, Steinberg W, Hellström AC, Andersson S, Hellman U, Auer G (2009) Differential tissue-specific protein markers of vaginal carcinoma. Br J Cancer 21: 1303–131410.1038/sj.bjc.6604975PMC267654119367286

[bib25] Hellman K, Alaiya AA, Schedvins K, Steinberg W, Hellström AC, Auer G (2004) Protein expression patterns in primary carcinoma of the vagina. Br J Cancer 91: 319–3261519938910.1038/sj.bjc.6601944PMC2409807

[bib26] Kulasingam V, Diamandis EP (2008) Strategies for discovering novel cancer biomarkers through utilization of emerging technologies. Nat Clin Pract Oncol 5: 588–5991869571110.1038/ncponc1187

[bib27] Lomnytska M, Becker S, Hellman K, Hellström A-C, Souchelnytskyi S, Mints M, Hellman U, Andersson S, Auer G (2010) Diagnostic marker protein patterns in squamous cervical cancer. Proteomics Clin Applications 4: 17–3110.1002/prca.20090008621137014

[bib28] Melsheimer P, Vinokurova S, Wentzensen N, Bastert G, von Knebel Doeberitz M (2004) DNA aneuploidy and integration of human papillomavirus type 16 E6/E7 oncogenes in intraepithelial neoplasia and invasive squamous cell carcinoma of the cervix uteri. Clin Can Res 10: 3059–306310.1158/1078-0432.ccr-03-056515131043

[bib29] Munoz N, Bosch FX, de Sanjose S, Herrero R, Castellsague X, Shah KV, Snijders PJ, Meijer CJ (2003) International agency for research on cancer multicenter cervical cancer study group. Epidemiologic classification of human papillomavirus types associated with cervical cancer. N Engl J Med 348: 518–5271257125910.1056/NEJMoa021641

[bib30] Näslund I, Auer G, Pettersson F, Sjövall K (1986) Evaluation of the pulse wash sampling technique for screening of uterine cervical carcinoma. Acta Radiol Oncol 25: 131–136301295710.3109/02841868609136391

[bib31] Nobbenhuis MA, Walboomers JM, Helmerhorst TJ, Rozendaal L, Remmink AJ, Risse EK, van der Linden HC, Voorhorst FJ, Kenemans P, Meijer CJ (1999) Relation of human papillomavirus status to cervical lesions and consequences for cervical-cancer screening: a prospective study. Lancet 3: 20–2510.1016/S0140-6736(98)12490-X10406360

[bib32] Noh DY, Ahn SJ, Lee RA, Kim SW, Park IA, Chae HZ (2001) Overexpression of peroxiredoxin in human breast cancer. Anticancer Res 21: 2085–209011497302

[bib33] Ono A, Kumai T, Koizumi H, Nishikawa H, Kobayashi S, Tadokoro M (2009) Overexpression of heat shock protein 27 in squamous cell carcinoma of the uterine cervix: a proteomic analysis using archival formalin-fixed, paraffin-embedded tissues. Hum Pathol 40: 41–491875549910.1016/j.humpath.2008.06.010

[bib34] Papanicolaou GN (1928) New cancer diagnosis. Proceedings of the Third Race Betterment Conference, pp 528–534

[bib35] Park JH, Kim YS, Lee HL, Shim JY, Lee KS, Oh YJ, Shin SS, Choi YH, Park KJ, Park RW, Hwang SC (2006) Expression of peroxiredoxin and thioredoxin in human lung cancer and paired normal lung. Respirology 11: 269–2751663508410.1111/j.1440-1843.2006.00849.x

[bib36] Singh M, Mehrotra S, Kalra N, Singh U, Shukla Y (2008) Correlation of DNA ploidy with progression of cervical cancer. J Cancer Epidemiol 2008: 1–710.1155/2008/298495PMC285893220445775

[bib37] Smith-Pearson PS, Kooshki M, Spitz DR, Poole LB, Zhao W, Robbins ME (2008) Decreasing peroxiredoxin II expression decreases glutathione, alters cell cycle distribution, and sensitizes glioma cells to ionizing radiation and H(2)O(2). Free Radic Biol Med 45: 1178–11891871852310.1016/j.freeradbiomed.2008.07.015PMC2628750

[bib38] Soini Y, Kallio JP, Hirvikoski P, Helin H, Kellokumpu-Lehtinen P, Kang SW, Tammela TL, Peltoniemi M, Martikainen PM, Kinnula VL (2006) Oxidative/nitrosative stress and peroxiredoxin 2 are associated with grade and prognosis of human renal carcinoma. APMIS 114: 329–3371672500810.1111/j.1600-0463.2006.apm_315.x

[bib39] Steinbeck RG, Auer G, Zetterberg AD (1999) Reliability and significance of DNA measurements in interphase nuclei and division figures in histological sections. Eur J Cancer 35: 787–7951050504110.1016/s0959-8049(98)00427-4

[bib40] Strzelecka-Kiliszek A, Buszewska ME, Podszywalow-Bartnicka P, Pikula S, Otulak K, Buchet R, Bandorowicz-Pikula J (2008) Calcium- and pH-dependent localization of annexin A6 isoforms in Balb/3T3 fibroblasts reflecting their potential participation in vesicular transport. J Cell Biochem 104: 418–4341804471610.1002/jcb.21632

[bib41] Sztolsztener ME, Strzelecka-Kiliszek A, Pikula S, Tylki-Szymanska A, Bandorowicz-Pikula J (2009) Cholesterol as a factor regulating intracellular localization of annexin A6 in Niemann-Pick type C human skin fibroblasts. Arch Biochem Biophys 15: 221–23310.1016/j.abb.2009.11.00119900398

[bib42] Van den IJssel P, Wheelock R, Prescott A, Russell P, Quinlan RA (2003) Nuclear speckle localisation of the small heat shock protein B-crystallin and its inhibition by the R120G cardiomyopathy-linked mutation. Exp Cell Res 287: 249–2611283728110.1016/s0014-4827(03)00092-2

[bib43] Wallin KL, Wiklund F, Angstrom T, Bergman F, Stendahl U, Wadell G, Hallmans G, Dillner J (1999) Type-specific persistence of human papillomavirus DNA before the development of invasive cervical cancer. N Engl J Med 341: 1633–16381057215010.1056/NEJM199911253412201

[bib44] Zhu X, Lv J, Yu L, Zhu X, Wu J, Zou S, Jiang S (2009) Proteomic identification of differentially-expressed proteins in squamous cervical cancer. Gynecol Oncol 112: 248–2561900797110.1016/j.ygyno.2008.09.045

[bib45] Zur Hausen H (2009) Papillomaviruses in the causation of human cancers-a brief historical account. Virology 384: 260–2651913522210.1016/j.virol.2008.11.046

